# Sub-lethal doses of Nucleopolyhedrosis Virus and synthetic ınsecticides alter the biological parameters of *Helicoverpa armigera* Hübner (Lepidoptera: Noctuidae)

**DOI:** 10.1371/journal.pone.0259867

**Published:** 2021-12-02

**Authors:** Allah Dita Abid, Syed Muhammad Zaka, Shafqat Saeed, Naeem Iqbal, Muhammad Nadir Naqqash, Muhammad Sohail Shahzad

**Affiliations:** 1 Department of Entomology, Bahauddin Zakariya University, Multan, Pakistan; 2 Department of Plant Protection, Ministry of National Food Security and Research, Islamabad, Pakistan; 3 Institute of Plant Protection, Muhammad Nawaz Sharif University of Agriculture Multan, Multan, Pakistan; King Khalid University, SAUDI ARABIA

## Abstract

Resistance management is very important for devising control strategies of polyphagous insect-pests like *Helicoverpa armigera* Hübner (Lepidoptera: Noctuidae). Considering the importance of resistance management, demographic features of selected and unselected populations of *H*. *armigera* were studied in 6 different treatments viz. emamectin benzoate, *Helicoverpa armigera* Nucleopolyhedrosis Virus (HaNPV), emamectin benzoate+HaNPV, spinetoram, spinetoram+HaNPV and control. Higher values for fecundity, intrinsic rate, the finite rate of increase (*λ*) were recorded in the control of selected as compared to the rest of treatment. Similarly, higher values for these population parameters viz. oviposition days, fecundity, intrinsic rate, the finite rate of increase were calculated in the unselected control. Similarly, net reproductive rate (*R*_*0*_) for selected and unselected control was higher as compared to the rest of the treatments. It may happen because these kinds of selection pressures can result in decreased fitness of the test insect thus decreased fitness of *H*. *armigera* in different treatments was observed as compared to the control. Additionally, quicker development of susceptible insects was observed because susceptible insects were growing without any stressor (xenobiotics) as compared to the rest which contributed to their faster development.

## Introduction

American bollworm (ABW), *Helicoverpa armigera* Hübner (Lepidoptera: Noctuidae), is one of the important pest attacks to a range of agricultural crops, such as fiber crops, horticultural plants, and vegetables [1–3]. In Pakistan, it has been considered the most dangerous and yield decliner of field crops from 1990s to early 21^st^ century [4]. Additionally, polyphagous nature, several generations, high fertility rate, migratory behavior, and development of resistance are among the important reasons that have made this pest very destructive [5, 6]. Annual losses of around 3 billion USD have been reported due to its attack [7].

Farmers in developing countries rely on chemical insecticides for the management of *H*. *armigera*. Continuous dependence on insecticides has resulted in insecticide resistance to approximately all major groups of insecticides in this notorious pest [8]. Therefore, insecticide resistance management activities by adding biocontrol agents like Nucleopolyhedrosis viruses (NPVs) in the control program are of primary importance to decrease insecticide usage and delaying the onset of resistance in insect pests which may lead to economic control of insect pests and better crop yield. NPVs can partly or completely replace the synthetic insecticides owing to their specificity and ecofriendly nature [9]. The NPVs are members of the Baculoviridae family (BV), which has been shown to be effective against a wide range of pests of forests and economically important crops [10]. This family includes two genera, the NPV and Granuloviruses (GV) [11].

Spinetoram is primarily a stomach poison with some contact toxicity. It is a mixture of two spinosyns A and D and is obtained from soil actinomycete *Saccharopolyspora spinosa* Mertz and Yao (Actinomycetales: Pseudonocardiaceae) after fermentation [12]. Spinetoram targets the binding sites on nicotinic acetylcholine receptors (nAChRs) and GABA receptors of insect nervous system [13]. After exposure to spinetoram, the insect stops feeding followed by paralysis and death. It is usually used against Lepidopteran and Dipteran, but its novel mode of action makes it relatively safer for non-target organisms and environment [14, 15]. Emamectin benzoate is a mixture of avermectins containing about 80% avermectin B1a and 20% avermectin B1b and is produced after fermentation of soil bacterium *Streptomyces avermitilis* [16, 17]. Emamectin benzoate is a selective insecticide, acaricide and nematicide which kills the target organisms by disrupting γ-aminobutyric acid (GABA) gated chloride channels, glutamate-gated chloride channel and other chlorine channels in nervous system [18]. Due to harsh environmental conditions of sub-tropical regions like Pakistan, NPV alone can’t be much effective. So, there is need of exploring the potential of NPV along with safer insecticides. Toxicity alone doesn’t give complete information regarding the use of any control strategy. In this regard, life table is important for ecologists, researchers, and pest managers since it provide better understanding of insect-pest ecology. It can be utilized in various studies involving insect ecology, physiology, and insecticides’ susceptibility [19–22].

Ignoring male population and stage differentiation are the biggest drawback of female-based age-specific life table analysis [23, 24]. So, female-based life tables can be erroneous and misguiding due to errors in results of important population parameters like growth, survival, and stage differentiation [9, 10, 15]. Fitness costs can occur in insects and include reduced survival and fecundity in the presence of pathogens [25, 26]. In order to determine if single or co-infection of control agents could affect the life traits such as fecundity, hatching and intrinsic rate of population increase. Two different questions were addressed in these series of experiments. How environmental changes such as insecticide treatments influence the dynamics of intrinsic rate of population of increase. The second question was: Is it possible to detect a cost associated with pathogens or combination of pathogen and insecticides. Age-stage, two-sex life table gave a solution to these shortcomings by taking these aspects viz. stage differentiation along with male population into consideration. It was developed by Chi and Liu [27] which was further refined by Chi and Getz [28]. Age-stage, two-sex life table have gained special attention of researchers [29, 30]. Considering the importance of resistance management and age-stage two sex life table analysis, demographic features of 12 different *H*. *armigera* populations were studied under different stress conditions.

## Materials and method

### Insect rearing and treatments

The emamectin benzoate selected and un-selected populations were obtained from a laboratory colony maintained at Institute of Pure and Applied Biology, Bahauddin Zakariya University, Multan, Pakistan. The larvae were reared on artificial diet [31] mentioned in Table 1. Adults of *H*. *armigera* were reared on honey and yeast solution. The treatments include spinetoram, emamectin benzoate and *Helicoverpa armigera* Nucleopolyhedrosis Virus (HaNPV) used alone and in combinations. Commercial formulations of spinetoram (Radiant^®^ 120 SC Arysta LifeScience Pakistan) and emamectin benzoate (Proclaim^®^ 019 EC, Syngenta Pakistan) were purchased from local market. However, HaNPV was used from laboratory maintained culture.

**Table 1:** Ingredients of artificial diet for rearing of *H*. *armigera* larvae.

Component	Quantity
Chickpea flour	100 g*
Yeast	30 g
Wesson’s salt mix	7 g
Methyl Paraben	2 g
Sorbic acid	1 g
Ascorbic acid	3 g
Agar	13 g
Vanderzant vitamin solution	8 ml**
Streptomycin sulphate	40 mg
Carbendazim	675 mg
Formalin	2 ml***
Water	720 ml

* Whole chickpea seeds could also be used (soak in distilled water overnight).

**28% solution in distilled water.

***not included in diets used for inoculation of larvae with virus and post-inoculation rearing.

To test a hypothesis if a single factor created three subpopulations having fitness cost compared with unselected and laboratory standard populations fecundity, developmental and survival rate; selected and unselected lines in the presence or absence of selection agent was studied as described previously [26, 32].

### Sub-lethal treatments and trans-generational effect

The sub-lethal doses (LC_25_) of HaNPV (0.32×10^9^) spinetoram (192.39 mg/l), emamectin benzoate (834.32 mg/l), spinetoram+HaNPV (0.25×10^9^ PIB/ml, 129.51mg/l), emamectin benzoate+HaNPV (0.25 PIB/ml ×10^9^, 890.09 mg/l) and untreated control were used based on previous published study of Abid et al. [33]. For this purpose, 200 second instar larvae of each of emamectin benzoate selected and un-selected population were exposed to sub-lethal doses of each treatment separately in petridishes containing treated diet. The larvae were allowed to feed on treated diet for three days and after that the surviving larvae were shifted to insecticide free artificial diet until pupation. The pupae were shifted to small plastic jars (0.5 liter) individually until emergence. After emergence, five pairs of adults of same age and group were paired randomly in plastic jars (05 liter). These groups were fed on 10% honey and yeast solution.

Transgenerational effects of these treatments were studied in the respective treatments. A total of 50 eggs were randomly selected from the progeny of each treatment for life table studies. Demographic features of *H*. *armigera* i.e., developmental time of eggs, larvae, pupae, those dying before adult stages, sexes (male and female), adults and female daily fecundity were recorded according to the age-stage two-sex life table theory [27, 28, 34] and analyzed using TWOSEX-MSChart [35]. According to the age-stage, two-sex life table theory [27], the age-specific survival rate (*l*_*x*_) and the age specific fecundity of the population (*m*_*x*_) are calculated as follows:

$$l_{x}=\sum_{j=1}^{m}s_{xj}$$ (1)

$$m_{x}=\frac{\sum_{j=1}^{m}s_{xj}f_{xj}}{\sum_{j=1}^{m}s_{xj}}$$ (2)

where, *m* is the number of stages of the study cohort.

The intrinsic rate of increase (*r*) which is defined as “the rate of increase per head under specified physical conditions, in an unlimited environment where the effects of increasing density do not need to be considered” was calculated by using the iterative bisection method from the Euler–Lotka formula [36] with age indexed from 0 (age of the newly laid eggs) as follows;

$$\sum_{x=0}^{\infty }e^{-r(x+1)}l_{x}m_{x}=1$$ (3)

The finite rate of increase (*λ;* the rate of increase per individual per unit time.) is calculated as follows [36];

$$\lambda =e^{r}$$ (4)

The mean generation time (*T*; the length of time that a population requires to increase to the *R*_*0*_-fold of its size at the stable age-stage distribution) was calculated as follows [36];

$$T=\frac{\ln R_{0}}{r}$$ (5)

As the insects were reared in groups, the number of individuals that survived to age “*x”* for each stage were recorded. The survival rate (*s*_*xj*_) to each age-stage unit was calculated as

$$s_{xj}=\frac{n_{xj}}{n_{01}}$$ (6)

where “*n*_*01*_*”* (the number of eggs used at the beginning of life table study) and “*n*_*xj*_*”* (the number of insects that survived to age *x* and stage *j*). Since we observed and collected the total number of eggs (*E*_*x*_) laid by all female adults together (the seventh life stage) at age *x*, female age-specific fecundity “*f*_*x7*_*”* and the net reproductive rate (*R*_*0*_) was calculated as Chang et al., [37].

$$f_{x7}=\frac{E_{x}}{n_{x7}}$$ (7)

$$R_{0}=\sum_{x=0}^{\infty }\sum_{j=1}^{k}s_{xj}f_{xj}$$ (8)

where “*k*” is the number of life stages.

Life expectancy another parameter which is defined by Shryock et al. [38] as “the average time that a member of a population is predictive to live”.

The age-specific life expectancy (*e*_*x*_) the time that individuals of age *x* are predictable to live for group rearing method 20 is calculated as;

$$e_{x}=\frac{\sum_{i=x}^{n}l_{i}}{l_{x}}$$ (9)

*l*_*i*_ = the probability that an individual of age *0* will survive to age *i*.

The bootstrap technique as described previously for individual reared method was used to estimate the standard errors for population parameters. All data calculated for each group was subjected to the bootstrap method with 10,000 resampling for estimating the standard errors of population parameters. Difference between treatments was then compared by using the paired bootstrap method [39, 40].

## Results

### Basic parameters

The basic parameters viz. pre-adult duration, adult duration, adult longevity, fecundity, oviposition period, Total pre-oviposition period (TPOP) and Adult pre-oviposition period (APOP) varied significantly among the treatments of both populations i.e. unselected and selected population are shown in Table 2.

**Table 2:** Effect of HaNPV, insecticides and their combinations on emamectin benzoate selected and unselected population of *Helicoverpa armigera*.

Parameter	Selected						Unselected					
	CT	Ema	HaNPV	HaNPV+ Ema	HaNPV+ Spine	Spine	CT	Ema	HaNPV	HaNPV+ Ema	HaNPV+ Spine	Spine
Pre-adult duration	25.51±0.09d	25.57±8.65cd	25.92±0.16c	27.97±0.29a	26.31±0.26b	26.53±0.12b	24.22±0.12a	23.22±0.16ab	20.50±0.14c	22.49±0.22b	20.96±0.41c	21.99±0.29c
Adult duration	8.96±0.22c	8.91±0.22c	8.48±0.10d	9.58±0.59b	10.31±0.27a	9.76±0.16b	12.22±0.25a	9.07±0.36c	10.50±0.34b	12.62±0.53a	10.65±0.62ab	11.56±0.24a
Female longevity	34.23±0.42b	34.24±0.42b	34.36±0.28b	37.00±1.07a	36.00±0.00a	36.11±0.31a	36.88±0.41a	32.50± 1.14c	31.71±0.52c	33.99±0.93b	31.66±0.31c	33.19± 0.58b
Male longevity	34.74±0.37b	34.75±0.37b	34.45±0.31b	33.52±12.95ab	23.95±18.34ab	36.49±0.66a	35.93±0.50a	27.76±10.86a	30.26±0.89a	34.69±0.54a	27.35±10.69a	33.48±4.22a
Adult pre-oviposition period	2.53±0.12b	2.47±0.12b	2.14±0.20b	1.33±0.31c	3.00±0.00a	1.44±0.18c	1.88±0.17b	1.99±0.76ab	2.57±0.20a	2.67±0.31a	2.67±0.31a	3.40±0.40a
Total pre-oviposition period	28.00±0.00b	28.00±0.00b	28.00±0.00b	29.00±0.00a	29.00±0.00a	28.00±0.00b	26.00±0.05a	25.00±0.00b	23.00±0.35c	25.00±0.23b	23.00±0.21c	25.00±0.00b
Oviposition days	6.18±0.39b	6.23±0.29b	6.36±0.29b	7.33±0.62a	7.00±0.00a	7.67±0.17a	8.41±0.12a	7.50±1.13b	8.14±0.26a	8.00±0.00a	8.00±0.00a	7.60±0.24b
Fecundity	337.63±29.10a	293.54±23.64ab	212.24±9.26c	258.64±10.68b	259.00±0.00b	230.88±1.78c	327.17±0.26b	400.95±46.28a	386.85±3.84a	377.66±0.31a	352.00±0.53b	409.39±2.75a

CT = control; Ema = Emamectin benzoate; HaNPV: *Helicoverpa armigera Nucleopolyhedrosisvirus;* Spine: Spinetoram

Lettering in rows is showing significant difference; Values are compared for selected and unselected population separately

In emamectin benzoate-selected population, pre-adult duration was significantly more i.e. 27.97 days in HaNPV+Emamectin benzoate treatment while it was lower in control i.e. 25.51 days. Adult duration was greater in HaNPV+spinetoram (10.31 days). While, lower adult longevity was calculated in HaNPV treatment with 8.48 days. Higher APOP and TPOP were 3.00 and 29.00 days in HaNPV+spinetoram treatment which decreased to minimum in spinetoram treatment i.e. 1.44 and 28.00 days, respectively. Oviposition period was significantly higher in spinetoram treatment (7.67 days). Significantly lower oviposition period was calculated in control with 6.18 days. Fecundity was more in control (337.63), while it was lower in HaNPV treatment (212.24).

In Unsel population, pre-adult duration was more in control (24.22 days) while it was lower in HaNPV treatment. Similarly, adult duration was greater in control with 12.22 days. While, lower adult duration was calculated in Emamectin benzoate treatment with 9.07 days. The TPOP was greater in control with 26.00 days and APOP (3.40 days) were higher in spinetoram. The TPOP decreased to minimum in HaNPV+spinetroam treatment with 23.00 days and APOP was minimum in control with 1.88 days. Oviposition period was significantly higher in control i.e. 8.41 days. Lower oviposition period was calculated in emamectin benzoate with 7.50 days. Fecundity was more in spinetoram treatment i.e. 409.39. While, fecundity was lower in control (327.17).

### Population parameters

Effects of different treatments viz. HaNPV alone, insecticides and combinations of insecticides with HaNPV and their respective control on life table parameters of *H*. *armigera* e.g. the intrinsic rate of increase (*r*), the finite rate of increase (*λ*), the net reproductive rate (*R*_*0*_), the mean generation time (*T*) and gross reproductive rate (*GRR*) reared in groups are shown in Table 3.

**Table 3:** Effect of HaNPV, insecticides and their combinations on emamectin benzoate selected and unselected population of *Helicoverpa armigera*.

Parameter	Selected						Unselected					
	CT	Ema	HaNPV	HaNPV+ Ema	HaNPV+ Spine	Spine	CT	Ema	HaNPV	HaNPV+ Ema	HaNPV+ Spine	Spine
The intrinsic rate of increase (*r)* per day	0.14±0.01a	0.09±0.01c	0.14±0.01a	0.08±0.02d	0.06±0.01d	0.12±0.02b	0.15±0.01a	0.09±0.01b	0.14±0.01a	0.10±0.02b	0.11±0.02b	0.12±0.02a
The finite rate of increase (*λ*) per day	1.16±0.01a	1.15±0.03	1.13±0.01a	1.08±0.02bc	1.06±0.01c	1.11±0.01b	1.17±0.01a	1.10±0.02b	1.15±0.02a	1.11±0.02b	1.11±0.02b	1.14±0.02a
The net reproductive rate (*R*_*0*_)	114.76±24.62a	99.76±21.07a	59.42±13.72b	16.29±8.24c	8.14±4.14c	41.60±12.52b	111.37±21.94a	18.43±10.06b	54.19±18.98b	23.73±11.97b	22.22±11.16b	41.13±17.17b
The mean generation time (*T*) in day	32.49±0.15c	32.50±0.13c	32.15±0.10c	33.01±0.12b	33.39±0.01a	32.57±0.03c	30.44±0.06a	29.75±0.02b	27.66±0.03c	29.68±0.02e	27.92±0.02f	29.22±2.60d

CT = control; Ema = Emamectin benzoate; NPV: Nucleopolyhedrosis virus; Spine: Spinetoram

Lettering in rows is showing significant difference; Values are compared for selected and unselected population separately

In the selected population, highest intrinsic rate of increase (*r*) and the finite rate of increase (*λ*) values were calculated in the control viz. 0.15 and 1.16 per day. While, lowest values of intrinsic rate of increase (*r*) and the finite rate of increase (*λ*) i.e. 0.06 and 1.06 per day were calculated in HaNPV+spinetoram treatment. Similarly, higher net reproductive rate i.e. *R*_*0*_ = 114.76 was also calculated in control. While, lower values 8.14 of *R*_*0*_ were observed in HaNPV+spinetoram treatment. Regarding mean generation time quicker development was observed in control as compared to the most effective treatment of HaNPV+spinetoram. Mean generation time (*T*) was higher in HaNPV+spinetoram treatment (33.39) while lower in control in 32.49 days.

In the Unselected population, higher population parameters like *r*, *λ*, *R*_*0*_ and *T* were 0.15, 1.17, 111.37 and 30.44, respectively were calculated in control. In the unselected population most effective treatment was emamectin benzoate. Lower values of *r* = 0.09, *λ* = 1.10, *R*_*0*_ = 18.43 and *T =* 29.75 were found in HaNPV+emamectin.

### Age-stage specific survival rate (*s*_*xj*_)

Calculated age-stage survival rates (*S*_*xj*_) of the selected and unselected population are given in Figs 1 and 2. Overlapping in *S*_*xj*_ curves indicates the variation in developmental rate between different individuals. Among the treatments of selected population, higher survival rate was observed in the control and emamectin benzoate treatment. While, only two individuals (one male and one female) successfully emerged from pupal stage. Where, female survived to 36 days while male survived to 37 days.

**Fig 1:** Effect of HaNPV, insecticides and their combinations on survival rate (*S*_*xj*_) on emamectin benzoate selected population of *Helicoverpa armigera*.

**Fig 2:** Effect of HaNPV, insecticides and their combinations on survival rate (*S*_*xj*_) on unselected population of *Helicoverpa armigera*.

Among the treatments of selected population, higher survival rate was observed in the control. Out of 50 eggs, 32 individuals successfully reached the adult stage. These male and female adults successfully managed to reach the age of maximum 38 days. While, only 3 individuals (1 male and 2 female) successfully emerged from pupal stage. Where, female survived to 35 days while male survived to 36 days.

### Age-stage life expectancy

The age-stage life expectancy (*e*_*xj*_), varied among the different treatments of two tested populations. The difference in the age-stage-specific life expectancy of two different CPB populations is shown in (Fig 3A and 3B). The life expectancy from age zero (*e*_*o*_) was maximum 41 days in the selected population, in treatment HaNPV+Emamectin benzoate. While, in unselected population was maximum 37 days were observed in the treatment HaNPV+Emamectin benzoate.

**Fig 3:** Effect of HaNPV, insecticides and their combinations on survival rate (*S*_*xj*_) on emamectin benzoate selected population (A) and Unselected population (B) of *Helicoverpa armigera*.

### Age-specific maternity (*l*_*x*_*m*_*x*_)

Age-specific survival rate (*l*_*x*_), age-specific fecundity of whole population (*m*_*x*_) and their product viz. age specific maternity (*l*_*x*_*m*_*x*_) of 6 treatments given to *H*. *armigera* populations are presented in Fig 4. In the selected population, age-stage specific fecundity (*f*_*x*_) approached the peak value of 160.28 on day 34. Lower peak viz. 50.35 was observed in HaNPV treatment on day 32. These graphs show that age-specific survival rate (*l*_*x*_) decreased gradually in the selected control than the rest of populations. The age-specific fecundity (*m*_*x*_) was higher in selected control viz. 30.14 while lowest value of 1.20 was observed in HaNPV+spinetoram treatment. For age-specific maternity (*l*_*x*_*m*_*x*_) the highest peak (19.90 offsprings/day) was observed on day 34 in the control while the lower peak value was only 0.048 offsprings/day in HaNPV+ spinetoram treatment.

**Fig 4:** Effect of HaNPV, insecticides and their combinations on age-stage specific survival (*l*_*x*_), age stage specific maternity (*m*_*x*_) and their product in emamectin benzoate selected population of *Helicoverpa armigera*.

In the unselected population, age-stage specific fecundity (*f*_*x*_) approached the peak value of 88.66 on day 30. Lower peak viz. 86.00 was observed in HaNPV+spinetoram treatment on day 28. These graphs show that age-specific survival rate (*l*_*x*_) decreased gradually in the unselected control than the rest of populations. The age-specific fecundity (*m*_*x*_) was higher in unselected control viz. 30.14 while lowest value of 3.80 was observed in emamectin benzoate treatment. For age-specific maternity (*l*_*x*_*m*_*x*_) the highest peak (19.28 offsprings/day) was observed on day 30 in the control while the lower peak value was only 0.30 offsprings/day in emamectin benzoate treatment (Fig 5).

**Fig 5:** Effect of HaNPV, insecticides and their combinations on age-stage specific survival (lx), age stage specific maternity (mx) and their product in emamectin benzoate selected population of *Helicoverpa armigera*.

## Discussion

Life table analysis is an effective tool for ecological studies and is used in assessment of growth, survival, reproductive capabilities as well as population projection of insects under varying conditions. Intrinsic rate (*r*) is assessed by age (*x*), the age-specific fecundity (*m*_*x*_) and the age-specific survival rate (*l*_*x*_) and of insect’s population and it helps us to forecast future population especially for insect pests and biocontrol agents [28]. Reproductive age of females and the peak value in reproductive age are the determining factors of growth rate of population and are also for forecasting future generations [41]. According to life table theory, the population increases only when *r* > 0 and net reproductive rate (*R*_*0*_) will be greater than 1 and the intrinsic rate of increase (*r*) is a more useful statistic than *R*_*0*_, to compare the population growth potential of various insect species [42, 43].

Higher fecundity (337.63 and 400.95 eggs) and optimum development time (24.22–25.51 days) was observed in control of both selected and unselected populations, respectively. These findings are comparable to the findings of Jaramillo et al. [44] who had reported that optimum conditions are key contributor towards optimum growth and faster multiplication of insects. In our case higher value of intrinsic rate and the finite rate of increase (*λ*) per day which were 0.15 and 1.16 per day, respectively, in control as compared to the rest of treatment. Similarly, higher value of net reproductive rate (*R*_*0*_) viz. 114.18 and 111.26 for selected and unselected control, respectively was calculated as compared to the control. These results are in accordance with Zaka et al. [45] and Abbas et al. [46] who have reported higher values for population parameters like *r*, *R*_*0*_, *λ* and others in susceptible and/or unselected population. It may happen since these kinds of selection pressures can result in decreased fitness of the test insect thus decreased fitness of *H*. *armigera* in different treatments was observed as compared to the control [47].

Similarly, higher survival rate for both controls was observed in selected and unselected populations. As a matter of fact, survival rate was higher in unselected control which is in accordance with the findings of Saddiq et al. [48]. Expected life expectancy was lesser in control as compared to HaNPV+Emamectin benzoate which showed higher life expectancy. These findings are comparable to the findings of Naqqash et al. [49] who have reported quicker development of susceptible insects as compared to the insects under constant pressure. When two or more bio-active agents are employed together, they synergize each other’s effectiveness and host spectrum while decreasing mortality time [50]. This could be due to the fact that the polyhedral bodies of NPV bind to the epithelium of the host and multiply, killing the gut cells. The midgut is the first binding site for POBs, where they multiply and then spread infection from cell to cell, killing the host. Resistance, on the other hand, decreases because of greater stress on the insect body [51]. Age-stage reproductive value of susceptible population was also higher in susceptible/unselected population as compared to the insects under constant pressure. These findings are comparable to the findings of Saeed et al. [47] who have reported higher reproductive value in control as compared to the insect under selection pressure.

## Conclusion

The population parameters were significantly affected by the selection pressure and insecticide+HaNPV treatments. So, according to this study a combination of HaNPV with spinetoram and emamectin benzoate can be more effective than separate treatments of HaNPV and insecticides.

## Supporting information

S1 Data (RAR)
